# CONSORT-epidural dexmedetomidine improves gastrointestinal motility after laparoscopic colonic resection compared with morphine

**DOI:** 10.1097/MD.0000000000011218

**Published:** 2018-06-22

**Authors:** Qiuxia Wan, Wengang Ding, Xiaoguang Cui, Xianzhang Zeng

**Affiliations:** Department of Anesthesiology, Second Hospital of Harbin Medical University, 246 Xuefu Road, Harbin, Heilongjiang, China.

**Keywords:** dexmedetomidine, gastrointestinal motility, laparoscopic colonic resection, thoracic epidural analgesia

## Abstract

**Background:**

We have previously shown that epidural dexmedetomidine, when used as an adjunct to levobupivacaine for control of postoperative pain after open colonic resection, improves recovery of gastrointestinal motility compared with morphine.

**Methods:**

Sixty patients undergoing laparoscopic colonic resection were enrolled and allocated randomly to treatment with dexmedetomidine (group D) or morphine (group M). Group D received an epidural loading dose of dexmedetomidine (5 mL, 0.5 μg/kg), followed by continuous epidural administration of dexmedetomidine (80 μg) in 0.125% levobupivacaine (240 mL) at a rate of 5 mL/h for 2 days. Group M received an epidural loading dose of morphine (5 mL, 0.03 mg/kg) followed by continuous epidural administration of morphine (4.5 mg) in 0.125% levobupivacaine (240 mL) at a rate of 5 mL/h for 2 days. Verbal rating score (VRS) of pain, postoperative analgesic requirements, side effects related to analgesia, and time to postoperative first flatus (FFL) and first feces (FFE) were recorded.

**Results:**

VRS and postoperative analgesic requirements were not significantly different between the treatment groups. In contrast, FFL and FFE were significant delayed in group M compared with group D (*P* < .05). Patients in group M also had a significantly higher incidence of nausea, vomiting, and pruritus (*P* < .05). No neurological deficits were observed in either group.

**Conclusions:**

Compared with morphine, epidural dexmedetomidine is a better adjunct to levobupivacaine for control of postoperative pain after laparoscopic colonic resection.

## 1 Introduction

Both the enhanced recovery after surgery (ERAS) protocol and laparoscopic surgery have been reported to be safe and effective for colorectal surgery and to result in shorter hospital stays, with earlier recovery of gastrointestinal motility.^[1–3]^ Despite these advantages of laparoscopic surgery, pneumoperitoneum, which is required for adequate visualization during laparoscopic surgery, has been reported to induce sympathetic activation and catecholamine release,^[4]^ thereby leading to the inhibition of gastrointestinal motility. Thoracic epidural analgesia is an effective method for the control of postoperative pain and is an important component of the ERAS protocol because it facilitates earlier out-of-bed mobilization and oral food intake, leading to shorter hospital stays and accelerated convalescence.^[5–8]^

Dexmedetomidine acts as an alpha-2 adrenergic agonist that was approved for intensive care unit sedation. We have previously shown that gastrointestinal motility recovers faster when epidural dexmedetomidine is used instead of morphine as an adjunct to levobupivacaine for control of postoperative pain after open colonic resection.^[9]^ Whether this beneficial effect also applies to laparoscopic surgery has not been determined, but we hypothesized that epidural dexmedetomidine should also provide benefits if used in combination with laparoscopic colonic resection. The primary efficacy endpoint of the study was time to postoperative first flatus (FFL), which is a variable that reflects gastrointestinal motility. Time to first feces (FFE) was used as a secondary endpoint. Time to FFL and FFE were compared for patients receiving different epidural analgesics for pain management.

## 2 Methods

### 2.1 Ethics approval

The research protocol was approved by the Ethics Committee of Harbin Medical University, Harbin, China (approval number: HMUIRB20140004) on March 3, 2014 (Chairperson Professor Mei Yin), and the study was registered in the Chinese Clinical Trial Registry (ChiCTR) (registration number ChiCTR-TRC-14004644) on May 14, 2014. Written informed consent was obtained from all study subjects.

### 2.2 Study subjects

Sixty patients, who met the American Society of Anaesthesiology Physical Status I/II criteria and were undergoing elective laparoscopic colonic resection in the Second Hospital of Harbin Medical University between December, 2014 and May, 2016, were enrolled in the study. Exclusion criteria were neurological or psychiatric disease, known allergy to local anesthetic agents, diabetes, a history of gastrointestinal motility disorders or prior abdominal surgery, renal or hepatic insufficiency, bleeding or coagulation abnormalities, and anticoagulant therapy. To eliminate possible confounding effects of different surgical techniques, all procedures were undertaken by a single surgeon who was experienced in performing laparoscopic colectomies. All colectomies were performed according to the protocol guidelines. Pneumoperitoneal and intracorporeal approaches were used to explore the abdomen, mobilize the colon, and identify critical structures. Patients received standardized care during the perioperative period and were allowed to drink small amounts of water during the first 24 hours after surgery. The patients were allowed to eat semisolid food 24 hours after surgery, but were not allowed to return to their normal diet until FFL occurred.

### 2.3 Treatment groups

Using a computer-generated random number table, the patients were randomly assigned to 1 of 2 groups and received different postoperative analgesia regimens when the surgeon closed the peritoneum. Patients allocated an odd number were assigned to the dexmedetomidine group (group D) and patients allocated an even number were assigned to the morphine group (group M). Patients in group D received an epidural loading dose of dexmedetomidine (5 mL, 0.5 μg/kg), followed by continuous epidural administration of dexmedetomidine (80 μg) in 0.125% levobupivacaine (240 mL) at a rate of 5 mL/h for 2 days. Patients in group M received an epidural loading dose of morphine (5 mL, 0.03 mg/kg), followed by continuous epidural administration of morphine (4.5 mg) in 0.125% levobupivacaine (240 mL) at a rate of 5 mL/h for 2 days.

### 2.4 Preparation for anesthesia

Basal pain threshold was expressed in terms of pain threshold (PTh) and pain tolerance threshold (PTTh), and postoperative pain was measured using an 11-point verbal rating score (VRS, 0–10). The method for measuring PTh and PTTh, and instructions for using the VRS, were explained to all patients. PTh and PTTh were measured by the microcurrent stimulation method, using an HD-EP-601C PTh detector (Hengaode Instrument Company Co, Ltd, Beijing, China) on the left upper arm. The detector generates a 50 Hz electrical stimulation, with a pulse width of 0.5 milliseconds. The intensity was increased gradually at a rate of 0.1 mA/s from 0 to 5 mA. The electrical PTh was reached when the patient first felt pain and the PTTh was reached when the patient felt that the pain was intolerable. The test was repeated after 10 minutes, and the average value of the 2 tests was calculated and recorded. All patients received midazolam (2.0 mg) and fentanyl (0.05 mg) intravenously (IV) 5 minutes before the baseline measurements and the epidural catheterization. Baseline measurements included heart rate, noninvasive arterial blood pressure, respiratory rate, peripheral oxygen saturation, and PTh and PTTh.

### 2.5 Implementation of anesthesia

An epidural catheter was placed in the T10/11 interspace, using a midline approach. The epidural space was identified by loss of resistance to saline and a test dose of 2% lignocaine with 1:200,000 adrenaline (3.0 mL) was administered to detect intrathecal or intravascular misplacement. After the test dose, 0.375% levobupivacaine was administered through the epidural catheter. When the level of sensory block was optimal, the patients underwent anesthetic induction and tracheal intubation after administration of propofol (2 mg/kg), fentanyl (3 μg/kg), and vecuronium (0.1 mg/kg). General anesthesia was maintained with 50% O_2_ containing 1.3% to 2.0% sevoflurane (2 L/min), using a semiclosed circle system. Muscle relaxation was maintained with vecuronium (0.1 mg/kg/h). Patients received 0.375% levobupivacaine (5 mL) at hourly intervals until the end of surgery. A central venous catheter was placed through the right subclavian vein for perioperative infusion and postoperative intravenous nutrition, as commonly performed at our institution. When the peritoneum was closed, a continuous infusor (Baxter) was attached to the epidural catheter for 48-hour postoperative pain control.

### 2.6 Assessments

To maintain blinding, the anesthetist who prepared the study solutions did not perform the epidurals and was not involved in patient management or assessments. The VRS was assessed at 2, 4, 6, 8, 16, 24, and 48 hours after surgery, both at rest and after coughing. Postoperative analgesic requirements were met with flurbiprofen (100 mg, IV), on request by the patient. The time to first analgesic dose and total analgesic dose were recorded. The time to postoperative FFL and FFE were recorded as the primary and second efficacy endpoints of the study. When FFL occurred within the first 6 hours after surgery, this was considered to reflect emptying of rectal gas rather than recovery of colonic transit, and the time to second flatus was recorded as the true time to recovery of colonic transit. Side effects attributable to dexmedetomidine and morphine, including bradycardia, hypotension, nausea and vomiting, and skin itching, were recorded. Hypotension was defined as mean arterial pressure <30% of baseline for 60 seconds, and bradycardia was defined as heart rate <50 beats/min. Neurological deficits, including pain, numbness, and lack strength were assessed 1, 2, 3, and 7 days after surgery to assess the safety of epidural dexmedetomidine.

### 2.7 Statistical analysis

The sample size was calculated by the power analysis performed using PASS 13.0 software (NCSS LLC). According to the result of FFL in our pilot study (means: group D, 31.3 hours; group M, 52.1 hours; SD 20.2 hours), in all, 54 patients were required to achieve a power of 90% and an α value of 0.05 for detection of differences between the 2 groups. Therefore, 60 participants (30 in each group) were enrolled in this study for the 10% possible dropouts. Statistical analyses of this study were performed using SPSS 19.0 software (IBM Corporation, Armonk, NY). The Kolmogorov–Smirnov test was used to test whether the data were normal distribution, and the chi-square test was used to analyze the incidence of complications, sex, and type of colectomy. The pain scores between groups were analyzed using the Mann–Whitney *U* test. Because of the normal distribution, the other variables were tested using an independent 2-sample *t* test. *P* < .05 was regarded as statistically significant.

## 3 Results

In all, 60 patients were randomly assigned to 1 of the 2 groups. One patient was withdrawn because of a previous gastrointestinal midline laparotomy, and 59 patients were, therefore, included in assessments of postoperative analgesic requirement and gastrointestinal motility. One patient from group D had mechanical bowel obstructions within the first 5 days, and, in group M, 1 patient had intraperitoneal bleeding and 1 patient was excluded because of epidural catheter blockage. In all, 56 patients thus completed the study. Baseline characteristics and surgical aspects did not differ significantly between the 2 groups (Table 1).

**Table 1:** Baseline characteristics and surgical aspects of the included patients in both the groups.

### 3.1 Postoperative pain control

At rest, the highest median VRS was 1 and the maximum interquartile range was 0 to 2 at all evaluation points for both groups, indicating satisfactory levels of pain control. There were no significant differences between group M and group D at any evaluation point. During coughing, VRS increased at most time points, although the highest median VRS score was 2 and the maximum interquartile range was 0 to 4 at all evaluation points for both groups, indicating the same satisfactory level of pain control. Comparison of groups M and D at each time point also showed no significant intergroup differences. Additionally, the time to first analgesic and total dose of analgesic were not significantly different between groups M and D (Table 2).

**Table 2:** Postoperative pain rating during 48 hours, the time to the first analgesic and total dose of analgesic in both the groups.

### 3.2 Recovery of gastrointestinal motility

The time to first postoperative passage of flatus was 30.2 ± 10.7 hours for group D (mean ± SD) and 38 ± 14.5 hours for group M (*P* < .05), and the 95% confidence interval (CI) was 4.4 to 21.8 hours. The time to first feces was 49.4 ± 12.5 hours for group D and 58.1 ± 17.1 hours for group M (*P* < .05) (Fig. 1), and the 95% CI was 4.1 to 36.9 hours. Group D thus demonstrated a significantly shorter time for recovery of gastrointestinal motility, using both primary and secondary study endpoints.

**Figure 1:** Time to postoperative first flatus and first feces of the 2 groups. Values are mean ± SD. D = dexmedetomidine, FFE = first feces, FFL = first flatus, M = morphine. ∗*P* < .05 compared with M group.

### 3.3 Postoperative side effects related to analgesic

Patients in group M had a higher incidence of nausea and vomiting and pruritus than patients in group D (Table 3; *P* < .05). In contrast, there were no significant differences in the incidence of bradycardia or hypotension between groups M and D. No patient in either group showed neurological deficits (Table 3).

**Table 3:** The comparison of postoperative side effects observed in both the groups.

## 4 Discussion

The present study showed a significant reduction of almost 8 hours in the time taken for return of gastrointestinal function after laparoscopic colectomy in patients who received epidural levobupivacaine combined with dexmedetomidine, compared with patients who received epidural levobupivacaine combined with morphine. This result is similar to that of our previous study, in which the same epidural anaesthetic management regimens were used after open colectomy.

Laparoscopic colorectal surgery is becoming the standard treatment for elective colorectal resection, and increased from 13.8% of all colorectal resections in 2007 to 42.6% in 2009.^[10]^ Many researchers have found that laparoscopic colorectal resection is associated with shorter hospital stays and lower morbidity, compared with open colectomy.^[11–13]^ The ERAS protocol was developed to enhance postoperative recovery for patients after open colorectal surgery, and has been widely adopted.^[14]^ A number of studies have shown that adoption of the ERAS protocol after laparoscopic colectomy leads to a significant reduction of postoperative hospitalization and a more rapid return of bowel function.^[15–17]^ However, the pneumoperitoneum which is required during laparoscopic surgery may induce sympathetic activation and catecholamine release, thereafter lead to the extended recovery time of gastrointestinal mobility after surgery.^[4]^

Co-administration of epidural morphine and local anesthetic is a common and effective method of postoperative pain control^[18]^ and an important component in the ERAS protocol. It is, however, well established that postoperative epidural morphine further reduces gastrointestinal motility,^[19–21]^ which is commonly impaired after intestinal surgery.^[22]^ An anesthetic that is suitable for epidural management of postoperative pain, and which does not impair gastrointestinal motility, would thus provide real clinical benefits.

Our previous study illustrated the beneficial effect of epidural dexmedetomidine on recovery of gastrointestinal motility when used as an adjunct to levobupivacaine for postoperative pain control after open colonic resection. The present study has confirmed that dexmedetomidine confers the same benefits after laparoscopic colectomy. Postoperative pain was well-controlled in both study groups, but patients in group D had a reduced incidence of nausea, vomiting, and pruritus compared with patients in group M.

The mechanism by which dexmedetomidine enhances gastrointestinal motility compared with morphine was not investigated in the present clinical study, but may be related to the dose and route of administration. A number of factors, including pain, the use of systemic opioid analgesia, increased sympathetic tone, and intestinal neuroinflammatory processes, have been reported to contribute to intestinal hypomotility.^[23]^ Dexmedetomidine acts on central α_2_-adrenoceptors, suppresses norepinephrine transporter function, and, via negative feedback, inhibits release of norepinephrine,^[24]^ thereby reducing sympathetic tone. Dexmedetomidine has also been shown to attenuate inflammatory response in rats suffering from intestinal injury.^[25]^ All of these effects may help dexmedetomidine to improve gastrointestinal motility. If, however, dexmedetomidine acted on gastric antrum α_2_-adrenoceptors, it would reduce secretion of acetylcholine via presynaptic inhibitory effects, which has been shown to inhibit gastrointestinal motility.^[26]^ It has also been suggested that both early and late components of postoperative gastric ileus are mediated via adrenergic pathways. Celiac ganglionectomy has been shown to improve impaired gastric motility induced by intestinal manipulation. Since celiac ganglionectomy removes the peripheral component of adrenergic neurons; this suggests that the peripheral sympathetic pathway mediates impaired gastric motility after surgery.^[22,27]^ For these reasons, we speculate that the ultimate effect of dexmedetomidine on gastrointestinal motility may be determined by the combined effect of activation of central and peripheral α_2_-adrenoceptors. In addition, a clinical study demonstrated that dexmedetomidine can decrease the postoperative serum diamine oxidase and intestinal fatty acid-binding protein expression significantly, indicating that dexmedetomidine might benefit the intestinal mucosa barrier function which may be an aspect for gastrointestinal motility.^[28]^

In addition, we speculated that the low dose of dexmedetomidine used in our study may partly contribute to the final results of gastrointestinal motility. The data from 2 previous clinical studies supported our speculation. The gastric emptying and gastrointestinal transit of patients were significantly inhibited when the total dose of dexmedetomidine infusion was almost 3.1 μg/kg.^[29]^ However, the delayed gastric emptying was normalized when the total dose was reduced to 1.0 μg/kg.^[30]^

The possible neurotoxicity effect of the low pH of dexmedetomidine solution, which was demonstrated by a previous animal study,^[31]^ has been discredited.^[32]^ None of the patients suffered from neurologic deficits in the present study, consistent with the results of previous clinical studies using peripheral, intrathecal, or epidural injections of dexmedetomidine.^[33–41]^ In contrast, there may be protective effect of epidural dexmedetomidine against neural cell death induced by lidocaine.^[42]^ Therefore, although large-scale studies are still needed, epidural dexmedetomidine appears to be both safe and efficacious.

## 5 Conclusion

Although we did not investigate the mechanisms by which dexmedetomidine affects gastrointestinal motility, the present study allows us to conclude that epidural dexmedetomidine is a better adjunct to levobupivacaine than morphine for the control of postoperative pain.

## Author contributions

**Conceptualization:** Qiuxia Wan.

**Data curation:** Qiuxia Wan, Wengang Ding, Xianzhang Zeng.

**Formal analysis:** Qiuxia Wan, Xianzhang Zeng.

**Funding acquisition:** Xianzhang Zeng.

**Investigation:** Qiuxia Wan.

**Project administration:** Qiuxia Wan, Xianzhang Zeng.

**Resources:** Qiuxia Wan.

**Software:** Xiaoguang Cui.

**Visualization:** Wengang Ding.

**Writing – original draft:** Qiuxia Wan, Wengang Ding, Xiaoguang Cui, Xianzhang Zeng.

**Writing – review & editing:** Qiuxia Wan, Xiaoguang Cui, Xianzhang Zeng.
